The article "Effect of Whole-Course Continuous Nursing Intervention Combined with a Nursing Practice Teaching Method on Quality of Life of Children with Functional Dyspepsia and Parents' Satisfaction Based on Smart Health" was published in 2022. Journal: J Healthc Eng.

# Effect of Whole-Course Continuous Nursing Intervention Combined with a Nursing Practice Teaching Method on Quality of Life of Children with Functional Dyspepsia and Parents' Satisfaction Based on Smart Health

**DOI:** 10.1155/2022/8638564

**Published:** 2022-02-16

**Authors:** Yue Li, Fenqin Xu, Jun Sun, Kangwei Mao, Suyun Sun, Jie Dai

**Affiliations:** ^1^Pediatric Internal Medicine Nursing Unit, The First People's Hospital of Lianyungang, The First Affiliated Hospital of Kangda College of Nanjing Medical University (The First People's Hospital of Lianyungang), Lianyungang 222000, Jiangsu, China; ^2^Nursing Department, The First People's Hospital of Lianyungang, The First Affiliated Hospital of Kangda College of Nanjing Medical University (The First People's Hospital of Lianyungang), Lianyungang 222000, Jiangsu, China; ^3^Department of Pediatrics, The First People's Hospital of Lianyungang, Lianyungang 222000, Jiangsu, China; ^4^Nursing Unit of Department of Neonatology, The First People's Hospital of Lianyungang, The First Affiliated Hospital of Kangda College of Nanjing Medical University (The First People's Hospital of Lianyungang, Lianyungang 222000, Jiangsu, China

## Abstract

With the development of information technology, it has become a part of people's lives. WeChat is not only a popular chatting tool in daily life but can also be used in the medical field. Functional dyspepsia is a common pediatric disease, with complex pathogenic factors, which are usually attributed to abnormal gastric acid secretion and gastrointestinal dysfunction. In our research, we aim to investigate the effects of whole-course continuous nursing intervention combined with a nursing practice teaching method on the quality of life (QOL) of children with functional dyspepsia and parents' satisfaction. One hundred and twenty children with functional dyspepsia admitted to our hospital (February 2019–February 2020) were retrospectively analyzed and equally divided into the experimental group (EG) and the control group (CG) according to the order of admission. The CG received whole-course continuous nursing intervention, and the EG received whole-course continuous nursing intervention combined with the nursing practice teaching method. Children's psychological states and QOL and parents' satisfaction of both groups were compared. After discharge, compared with the CG, the negative emotion scores in the EG were remarkably lower (*P* < 0.001). After discharge, compared with the CG, the QOL scores (*P* < 0.001), the proportion of children with good and excellent QOL (*P* < 0.05), and parents' satisfaction (*P* < 0.001) in the EG were remarkably higher. For children with functional dyspepsia, whole-course continuous nursing intervention combined with the nursing practice teaching method can improve their negative emotions, QOL, and parents' satisfaction, which should be popularized in practice.

## 1. Introduction

Children often present with abdominal pain, abdominal distension, nausea, and vomiting, and some of them are also complicated with neurosis, anxiety neurosis, and other mental problems [1, 2], which seriously affect their growth and development. It is reported that the incidence of functional dyspepsia accounts for 40% in the pediatric outpatient department in China [3]. Most of the children will get better with proper medication. However, due to their unchanged lifestyle after discharge, the disease can still be triggered by bad diet structure and psychological problems [4, 5]. In this way, the recurrence rate of functional dyspepsia in a clinic is high [6, 7], which poses a threat to children's physical and mental health. In order to reduce the recurrence rate of children after discharge, it is very important to take effective nursing measures. In practice, some scholars have applied whole-course continuous nursing intervention in children with gastric cancer and found that their quality of life (QOL) has been conspicuously improved within one year after discharge [8], which shows that this nursing mode can enhance the management efficiency and play the dual management role of psychology and physiology by focusing on the potential health problems of children [9]. Suffering from functional dyspepsia, the children have more severe negative emotions, together with poor treatment enthusiasm and gradually decreasing compliance after discharge [10, 11], which is not conducive to the recovery of the disease. Due to the poor compliance of children, giving them all-around quality nursing intervention during treatment has been a clinical consensus [12]. This kind of nursing mode coordinates with the intervention during hospitalization, which finally improves patients' QOL [13]. In this study, after the whole-course continuous nursing intervention, the psychological state of the two groups was improved. Previous studies show that the immune system and gastrointestinal system are controlled by the neuroendocrine system [14].

At present, as clinical experience is little, no application of whole-course continuous nursing intervention in children with functional dyspepsia has been found. Therefore, it is vital to choose the appropriate teaching method as the foundation. With constructivism as its core, the practice teaching method aims to integrate the theoretical knowledge of the whole-course continuous nursing intervention into practice, through which the nursing staff can improve their competency [15, 16]. In this paper, the actual effect of whole-course continuous nursing intervention combined with a nursing practice teaching method on children with functional dyspepsia was explored.

## 2. Materials and Methods

### 2.1. General Data

A retrospective analysis of the data of children with functional dyspepsia admitted to our hospital (February 2019–February 2020) was conducted. The inclusion criteria were as follows: (1) Children's parents fully understood the research process and signed the consent form. (2) Children were diagnosed with functional dyspepsia by examination in accordance with *the Rome IV Criteria for the Diagnosis of Functional Gastrointestinal Disorders in Children* [17]. (3) Children were under the age of 10. (4) Children were diagnosed for the first time. The exclusion criteria were as follows: (1) children who had mental problems or could not be communicated with [18]; (2) children who had other digestive diseases, diabetes mellitus, hyperthyroidism, hematological diseases, cardiovascular diseases, and organ dysfunction [19]; and (3) children who were with extremely poor treatment compliance [20].

A total of 120 children were included in this study and equally divided into the experimental group (EG) and the control group (CG) according to the order of admission. There was no statistical difference in the children's general data between the two groups (Table 1). The study was approved by the hospital's ethics committee.

### 2.2. Withdrawal Criteria

The withdrawal criteria were as follows: (1) Children who experienced adverse or serious adverse events were considered inappropriate to continue the experiment. (2) If children's conditions deteriorated during the experiment, it was considered inappropriate to continue to receive the experiment according to the doctor's judgment. (3) Children who had severe complications and special physiological changes were considered inappropriate to continue the experiment according to the doctor's judgment. (4) Children's parents who were unwilling to continue during the follow-up and asked the research group for a withdrawal from the clinical trial. The medical record sheets of the withdrawn cases were kept, but the data were not analyzed.

### 2.3. Methods

The CG was given whole-course continuous nursing intervention. The specific steps were as follows: (1) Nurses built the whole-course continuous nursing intervention group for parents of children with functional dyspepsia. The head nurse was set as the administrator, and then experts and nutrition professors acted as instructors to formulate the whole-course continuous nursing guiding strategies. Nursing staff ought to communicate with the parents at the children's admission to gain their trust and invite them into the WeChat group with the name “Department + Name + Bed Number” for better information collection and management. Nursing staff also popularized relevant knowledge in the group to help the parents master the right home nursing methods and to enrich their knowledge. The parents could communicate with each other in the group and ask about the children's condition. Then, nursing staff should answer the questions in time to help parents with home nursing, encourage them to share their children's recovery conditions in the group, and collect the information that could not be accessed in telephone follow-up so as to enhance the utilization efficiency of the WeChat group. (2) When the children were admitted to the hospital, the nursing staff mastered the children's information in detail and mapped out the nursing plans according to their actual situation. When the children were discharged, the nursing staff recorded the relevant information (children's name, contact information, family address, family members, and main family nursing staff) again, gave discharge guidance according to their recovery condition, and provided home nursing instruction handbooks. Children's parents were reminded to let children take acid-suppressive drugs and gastric mucosal protective agents on time, to feed gastroprokinetic drugs if children had a sense of fullness, to prepare soft clothes for keeping the abdomen warm, and to help children do physical exercise. Furthermore, due to the negative emotions in children with functional dyspepsia, children's parents were also informed about the importance of mental nursing, which was in need of conciliation in time. (3) The first telephone follow-up was conducted 3 days after discharge to see whether the children complied with the doctor's medication and had symptoms like abdominal pain and inappetence. Then, the telephone follow-up was once a week. One month after discharge, it was changed to once a month, which was for one year. (4) Children with severe symptoms should be hospitalized immediately. For children with special conditions, nursing staff should follow up for door-to-door diagnosis and treatment using the vehicles provided by the hospital, so as to solve problems for the children's parents. (5) Regular lectures on health education were organized, and billboards in communities were set up to improve family members' understanding of functional dyspepsia. The nursing staff updated the lecture information on the billboards, inviting the children and their families to join in for learning and improving the quality of home nursing.

The EG was given whole-course continuous nursing intervention combined with a nursing practice teaching method, that is, to add a nursing practice teaching method on the basis of the CG. The specific steps were as follows: (1) A workshop was set up, and the teaching plan was formulated by the teachers. The specific teaching plan was described as follows: Opening remarks (role play or actual case introduction) introduced the topic of continuous nursing. General information of nursing practice teaching was provided. Learning objectives were formulated to enable nurses to grasp the knowledge about continuous nursing. Problems related to continuous nursing, functional dyspepsia, and pediatric nursing were put forward. Each problem was analyzed by the teachers, and then new problems were put forward. The learning effects of nurses were investigated, and their ability to solve practical problems was evaluated. (2) Teachers should conduct role-play training for nurses before class to ensure that the scenario simulation can meet the expected requirements through which nurses can learn continuous nursing knowledge and apply it in practice. (3) Nurses should consult the relevant knowledge of continuous nursing and functional dyspepsia, analyze it combined with actual cases, put it into practice, and ask teachers about the problems in the next class, so as to improve their continuous nursing ability.

### 2.4. Observation Criteria

#### 2.4.1. Psychological State

It was evaluated according to the self-rating anxiety (SAS) scale and self-rating depression (SDS) scale [21]. Each of the scales included 20 items, with a total score of 100 points. Higher scores indicated more severe negative emotions in children. The scale was completed by the children's parents before nursing (*T*_1_), 3 months after discharge (*T*_2_), and 1 year after discharge (*T*_3_).

#### 2.4.2. QOL

It was evaluated according to the QOL scale for children and adolescents (QLSCA) [22]. The scale had 13 dimensions, such as self-satisfaction, teacher-student relationship, somatic feelings, peer relationship, parent-child relationship, exercise capacity, learning ability and attitude, self-concept, negative emotions, homework attitude, activity opportunistic, and life convenience, which formed 4 factors, namely, social psychological function, physical and mental health, living environment, and QOL satisfaction. The QLSCA score had 4 grades. 29 points and below indicated poor QOL, 30 to 59 points indicated medium QOL, 60 to 69 points indicated good QOL, and 70 points and above indicated excellent QOL. The scale was completed by the children's parents before nursing (*T*_1_), 3 months after discharge (*T*_2_), and 1 year after discharge (*T*_3_).

#### 2.4.3. Parents' Satisfaction

The self-made scale of our hospital was used to evaluate the total satisfaction of nursing and the satisfaction of health education, follow-up, online communication, and children's rehabilitation, with the score of each part being between 0 and 10 points. Higher scores indicated a higher degree of parents' satisfaction.

### 2.5. Statistical Processing

In this study, the data were processed by SPSS20.0 and graphed by GraphPad Prism7 (GraphPad Software, San Diego, USA). Including enumeration data and measurement data, the study used the *X*^2^ test and *t*-test. The differences were statistically significant at *P* < 0.05.

## 3. Results

### 3.1. Comparison of the Psychological State of Children

After discharge, compared with the CG, the negative emotion scores of the EG were conspicuously lower (*P* < 0.001) (Figure 1).

*Note.* In Figure 1, the abscissa from left to right was *T*_1_, *T*_2_, and *T*_3_, respectively. In the figure, the line with dots was the EG, and the line with squares was the CG. ^#^*P* < 0.001. Figure 1(a) was the SAS score. No obvious difference was found in the SAS scores at *T*_1_ between both groups (60.12 ± 2.41 vs 60.23 ± 2.32, *P* > 0.05). The SAS scores at *T*_2_ and *T*_3_ in the EG were obviously lower than those in the CG (39.65 ± 2.52 vs 44.68 ± 3.20 and 19.10 ± 2.65 vs 25.65 ± 2.10, *P* < 0.001). Figure 1(b) was the SDS score. No obvious difference was found in the SDS scores at *T*_1_ between both groups (62.65 ± 3.40 vs 62.54 ± 3.42, *P* > 0.05). The SDS scores at *T*_2_ and *T*_3_ in the EG were obviously lower than those in the CG (38.24 ± 3.20 vs 49.65 ± 3.22 and 19.87 ± 1.22 vs 27.62 ± 2.01, *P* < 0.001).

### 3.2. Comparison of QOL

After discharge, compared with the CG, the QOL scores (*P* < 0.001) and the proportion of children with good and excellent QOL (*P* < 0.05) in the EG were remarkably higher (Figures 2 and 3).

*Note.* In Figure 2, the abscissa from left to right was *T*_1_, *T*_2_, and *T*_3_, respectively, and the ordinate was QLSCA (points). In the figure, the black area was the EG, and the gray area was the CG. ^#^*P* < 0.001. No obvious difference was found in QLSCA scores at *T*_1_ between both groups (66.21 ± 5.65 vs 67.10 ± 5.47, *P* > 0.05). The QLSCA scores at *T*_2_ and *T*_3_ in the EG were obviously higher than those in the CG (88.65 ± 6.10 vs 70.68 ± 2.34 and 90.10 ± 6.41 vs 82.68 ± 6.15, *P* < 0.001).

*Note.* In Figure 3, the black area denotes poor QOL, the dark gray area denotes medium QOL, the light gray area indicates good QOL, and the white area indicates excellent QOL. In Figures 3(a)–3(c), the EG was on the left and the CG was on the right. Figure 3(a) shows the QOL at *T*_1_. The number of children with poor QOL, medium QOL, good QOL, and excellent QOL in the EG was 22 (36.7%), 30 (50.0%), 8 (13.3%), and 0 (0.0%), respectively, and that in the CG was 21 (35.0%), 32 (53.3%), 7 (11.7%), and 0 (0.0%), respectively, with no obvious difference between both groups (*P* > 0.05). Figure 3(b) shows the QOL at *T*_2_. The number of children with poor QOL, medium QOL, good QOL, and excellent QOL in the EG was 3 (5.0%), 24 (40.0%), 21 (35.0%), and 12 (20.0%), respectively, and that in the CG was 6 (10.0%), 36 (60.0%), 10 (16.7%), and 8 (13.3%), respectively. The number of children with good and excellent QOL in the EG was obviously higher than that in the CG (*P* < 0.05). Figure 3(c) shows the QOL at *T*_3_. The number of children with poor QOL, medium QOL, good QOL, and excellent QOL in the EG was 0 (0.0%), 15 (25.0%), 27 (45.0%), and 18 (30.0%), respectively, and that in the CG was 3 (5.0%), 23 (38.3%), 21 (35.0%), and 13 (21.7%), respectively. The number of children with good and excellent QOL in the EG was obviously higher than that in the CG (*P* < 0.05).

### 3.3. Comparison of Parents' Satisfaction

Compared with the CG, the satisfaction of parents in the EG was obviously higher (*P* < 0.001) (Table 2).

## 4. Discussion

Functional dyspepsia is a common disease in the pediatric digestive outpatient department, which is featured with a high recurrence rate, a long course of disease, and long-term treatment. The disease is usually caused by the abnormal secretion of gastrointestinal hormones. Some children are complicated with psychological problems. As we know, nursing intervention after discharge is helpful to improve the nutritional awareness of children and their parents, increase their disease cognition, and then decrease the recurrence rate. Continuous nursing is a common clinical nursing mode in recent years, which emphasizes more patients' potential health problems and the intervention of both physical and mental state. The negative emotions of children will affect their gastrointestinal function and even greatly impair their immunity. On the contrary, the alleviation of negative emotions indicates that the pathogenic factors of functional dyspepsia are reduced, the immunity is improved, and the disease is not easy to relapse.

However, it is not clear whether continuous nursing should be carried out for children after discharge. Some studies show that, after discharge, children still have bad eating habits and psychological problems [23, 24]. Long-term malnutrition seriously affects the physical and mental development of children. As the whole-course continuous nursing intervention has not been applied in children with functional dyspepsia before, this study especially took nursing practice teaching as the support, in which the nurses had a deeper cognition of functional dyspepsia. Scenario simulation teaching and case teaching enabled nurses to master the characteristics of the disease and children's mental activity.

Furthermore, nurses' perception, memory, and application abilities were fully improved, and they could clearly express themselves in health education and online communication, which yielded good results. The study showed that after discharge, compared with the CG, the negative emotion scores of the EG were obviously lower (*P* < 0.001). The reason is that the nursing staff experienced the emotional expressions of the children in the process of scenario simulation. Nurses put themselves in the place of children's parents to communicate with them, provided family nursing guidance from the perspective of children, and made full use of the active role of home nursing. The study carried out by El-Nagger N S et al., showed that the application of a practical teaching method in the nursing of children with pneumonia could comfort them and reduce their anxiety [25], which is consistent with the results of this study.

## 5. Conclusion

In our study, after one year's follow-up, compared with the CG, the scores of QOL in the EG were obviously higher (*P* < 0.05), and the proportion of children with good and excellent QOL was obviously higher (*P* < 0.05). The reason lies in that the nursing staff had paid more attention to humanistic care and professionalism through nursing practice teaching; therefore, the children's parents trusted more in nurses. One year after discharge, the children and their parents still had nursing compliance, and the recurrence rate of the disease was reduced. Therefore, compared with the CG, the satisfaction of children's parents in the EG was obviously higher (*P* < 0.001).

In conclusion, for children with functional dyspepsia, whole-course continuous nursing intervention combined with nursing practice teaching method can improve their negative emotions, QOL, and parents' satisfaction, which should be popularized in practice.

## Figures and Tables

**Figure 1:** Comparison of the psychological state of children (*x* ± *s*, points).

**Figure 2:** Comparison of QOL (*x* ± *s*, points).

**Figure 3:** Changes in QOL (*n* (%)).

**Table 1:** Comparison of general data.

Group	EG (*n* = 60)	CG (*n* = 60)	*X* ^2^/*t*	*P*
Gender			0.034	0.854
Male	34	33		
Female	26	27		
Age (years)				
Range	2–10	3–10		
Average age	5.21 ± 2.22	5.25 ± 2.10	0.101	0.919
Course of disease (weeks)				
Range	4–10	4–12		
Average age	7.65 ± 1.23	7.45 ± 1.24	0.887	0.377
Visit time (h)	2.65 ± 0.65	2.54 ± 0.67	0.913	0.363
Blood pressure				
Systolic blood pressure	120.65 ± 9.21	120.68 ± 9.22	0.018	0.986
Diastolic blood pressure	84.98 ± 7.98	84.96 ± 7.54	0.014	0.989
BMI (kg/m^2^)	22.10 ± 3.21	22.04 ± 3.10	0.104	0.917
Serum gastrin (pg/mL)	119.32 ± 20.12	119.54 ± 20.65	0.059	0.953
Serum motilin (pg/mL)	320.65 ± 30.14	320.68 ± 29.68	0.005	0.996
Somatostatin (pg/mL)	30.12 ± 3.65	30.58 ± 3.41	0.713	0.477
Residence			0.035	0.852
Urban	36	37		
Rural	24	23		
Parents' monthly income (yuan)			0.134	0.715
≥5000	32	30		
＜5000	28	30		
Parents' educational degree				
Middle school degree and below	12	14	0.196	0.658
Senior high school degree	26	28	0.135	0.714
University degree and above	22	18	0.600	0.439

**Table 2:** Comparison of parents' satisfaction (*x* ± *s*, points).

Group	EG (*n* = 60)	CG (*n* = 60)	*X* ^2^/*t*	*P*
Total nursing satisfaction	9.01 ± 0.54	8.21 ± 0.41	9.140	<0.001
Satisfaction of health education	9.23 ± 0.24	7.88 ± 0.34	25.127	<0.001
Satisfaction of follow-up	8.98 ± 0.50	7.64 ± 0.58	13.554	<0.001
Satisfaction of online communication	8.96 ± 0.42	8.12 ± 0.43	10.825	<0.001
Satisfaction of children's rehabilitation	9.21 ± 0.20	8.45 ± 0.34	14.924	<0.001

## Data Availability

The datasets used and/or analyzed during the current study are available from the corresponding author on reasonable request.

## References

[1] Chumpitazi B. P., Robayo-Torres C. C., Tsai C. M. (2018). Demographic and clinical correlates of mucosal disaccharidase deficiencies in children with functional dyspepsia. *Journal of Pediatric Gastroenterology and Nutrition*.

[2] Rui-Hua H. E. (2019). Effect of humanized nursing intervention on anxiety and quality of life in patients with functional dyspepsia. *Smart Healthcare*.

[3] Vivekanand S., Meenal S., Schurman J. V., Friesen C. A. (2018). Histopathological changes in the gastroduodenal mucosa of children with functional dyspepsia. *Pathology, Research & Practice*.

[4] Lei C., Paediatrics D. O. (2018). Analysis on the value of whole process nursing for children with acute dyspeptic diarrhea. *Journal of Mathematical Medicine*.

[5] Mokha J. S., Hyams J. S., Glidden N. C., Balarezo (2021). Characterizing clinical features and location:specific gene expression profiles associated with pain burden in children with functional dyspepsia. *Neuro-Gastroenterology and Motility*.

[6] Browne P. D., den Hollander B., Speksnijder E. M. (2019). Gut-directed hypnotherapy versus standard medical treatment for nausea in children with functional nausea or functional dyspepsia: protocol of a multicentre randomised trial. *BMJ Open*.

[7] Edwards T., Friesen C., Schurman J. V. (2018). Classification of pediatric functional gastrointestinal disorders related to abdominal pain using Rome III vs. Rome IV criterions. *BMC Gastroenterology*.

[8] Colman R. J., Rosario N., Analydia G. B. (2018). Functional GI disorders are prevalent among pediatric patients with persistent asthma: functional GI disorders and asthma. *Journal of Digestive Diseases*.

[9] Kumari M. V., Devanarayana N. M., Amarasiri L. (2018). Association between functional abdominal pain disorders and asthma in adolescents: a cross-sectional study. *World Journal of Clinical Cases*.

[10] Ibrahim A., Hamdy A. M., Elhodhod M. A. (2020). Prevalence of functional gastrointestinal disorders among school-aged children and adolescents, A multicenter study. *QJM: Monthly Journal of the Association of Physicians*.

[11] Rahmani P., Ghouran-Orimi A., Motamed F. (2020). Evaluating the effects of probiotics in pediatrics with recurrent abdominal pain. *Clinical and Experimental Pediatrics*.

[12] Belousova O. Y., Kazaryan L. V. (2019). Functional dyspepsia in children. Problems and prospects of symptomatic therapy. *Child`s Health*.

[13] Ivana T., Iva H. (2018). Initial diagnosis of functional gastrointestinal disorders in children increases a chance for resolution of symptoms. *Pediatric Gastroenterology Hepatology & Nutrition*.

[14] Goyal O., Nohria S., Dhaliwal A. S. (2020). Prevalence, overlap, and risk factors for Rome IV functional gastrointestinal disorders among college students in northern India. *Indian Journal of Gastroenterology*.

[15] Lalouni M., Ljótsson B., Bonnert M. (2018). Clinical and cost effectiveness of online cognitive behavioral therapy in children with functional abdominal pain disorders. *Clinical Gastroenterology and Hepatology*.

[16] Friesen C. A., Colombo J. M., Schurman J. V. (2019). The evolving role of mucosal histology in the evaluation of pediatric functional dyspepsia: a review. *Gastrointestinal Disorders*.

[17] Singh M., Singh V., Schurman J. V. (2020). Mucosal Th17 cells are increased in pediatric functional dyspepsia associated with chronic gastritis. *Digestive Diseases and Sciences*.

[18] Manoppo J., Somali R., Aspr P. (2020). Fecal calprotectin and its association with functional dyspepsia in children. *Paediatrica Indonesiana*.

[19] Galai T., Moran-Lev H., Cohen S. (2020). Higher prevalence of obesity among children with functional abdominal pain disorders. *BMC Pediatrics*.

[20] Ünlüsoy A. A., Yılmaz G., Eğritaş Ö. G. (2018). The effect of helicobacter pylori eradication on functional dyspepsia in turkish children. *Helicobacter*.

[21] Belmer S. V., Volynets G. V., Gorelov A. V. (2020). Functional digestive disorders in children. Guidelines of the spediatric ghn. *Rossiyskiy Vestnik Perinatologii i Pediatrii (Russian Bulletin of Perinatology and Pediatrics)*.

[22] Ipatov A. A., Ipatova M. G. (2021). Management of functional gastrointestinal disorders in children. Focus on restoring intestinal microenvironment and motility. *Meditsinskiy Sovet = Medical Council*.

[23] Spatuzzo M., Chiaretti A., Capossela L., Covino M., Gatto A. (2021). Abdominal Pain in Children: The Role of Possible Psychosocial Disorders. *European Review for Medical and Pharmacological Sciences*.

[24] Tambucci R., Quitadamo P., Ambrosi M., De P. (2018). Association between obesity/overweight and functional gastrointestinal disorders in children. *Journal of Pediatric Gastroenterology and Nutrition*.

[25] El-Nagger N. S., El-Sayed L. A. (2021). Vapevidence-based nursing practices for prevention of ventilator-associated pneumonia in pediatric intensive care units. *Evidence-Based Nursing Practices for Prevention of Ventilator-Associated Pneumonia in Pediatric Intensive Care Units*.

